The article "Long non-coding RNA LINC00152 promotes gallbladder cancer metastasis and epithelial–mesenchymal transition by regulating HIF-1α via miR-138" was retracted in 2023. Reasons: manipulated images; duplicated images; unreliable data; unreliable results or conclusions.

# Long non-coding RNA LINC00152 promotes gallbladder cancer metastasis and epithelial–mesenchymal transition by regulating HIF-1α via miR-138

**DOI:** 10.1098/rsob.160247

**Published:** 2017-01-11

**Authors:** Qiang Cai, Zhenqiang Wang, Shouhua Wang, Mingzhe Weng, Di Zhou, Chen Li, Jiandong Wang, Erzhen Chen, Zhiwei Quan

**Affiliations:** 1 Department of General Surgery, XinHua Hospital, Shanghai JiaoTong University School of Medicine, Shanghai 200092, People's Republic of China; 2 Shanghai Key Laboratory of Gastric Neoplasms, Department of Surgery, Shanghai Institute of Digestive Surgery, Ruijin Hospital, Shanghai JiaoTong University School of Medicine, Shanghai 200025, People's Republic of China; 3 Department of Emergency, Ruijin Hospital, Shanghai JiaoTong University School of Medicine, Shanghai 200025, People's Republic of China

**Keywords:** long non-coding RNA LINC00152, gallbladder cancer, metastasis, epithelial–mesenchymal transition, HIF-1α, miR-138

## Abstract

Long non-coding RNA LINC00152 had been reported as an oncogene in gastric and hepatocellular cancer. In this study, we show that LINC00152 is overexpressed in gallbladder cancer (GBC) tissue samples and cell lines. The high LINC00152 levels correlated negatively with the overall survival time in GBC patients. Functionally, LINC00152 dramatically promoted cell migration, invasion and epithelial–mesenchymal transition (EMT) progression *in vitro. In vivo*, LINC00152 overexpression significantly promoted tumour peritoneal spreading and metastasis. Mechanistic analyses indicated that LINC00152 functions as a molecular sponge for miR-138, which directly suppresses the expression of hypoxia inducible factor-1α (HIF-1α). We revealed that miR-138 is a suppressor of GBC cell metastasis and EMT progression, and a similar phenomenon was observed in HIF-1α knockdown NOZ cells. Through binding to miR-138, LINC00152 has an oncogenic effect on GBC. Overall, our study suggested that the LINC00152/miR-138/HIF-1α pathway potentiates the progression of GBC, and LINC00152 may be a novel therapeutic target.

## 1. Introduction

Gallbladder cancer (GBC) is the fifth most frequent gastrointestinal malignancy and one of the most lethal cancers worldwide [1]. Characterized by its early lymph node invasion and distant metastasis, GBC is usually diagnosed at its advanced stage and is then lacking effective therapies [2]. Taken all stages together, GBC has an overall 5-year survival of less than 5% and mean survival of less than six months [3]. Therefore, a better comprehending of the early events related to GBC metastasis is essential to reduce mortality.

One of the major mechanisms that facilitates tumour migration and invasion is the epithelial–mesenchymal transition (EMT), which is a process endowing epithelial cells with mesenchymal properties. The transdifferentiation is well characterized by reduced cell-to-cell adhesion and enhanced motility [4]. Accumulating evidence has shown that EMT plays an important role in GBC [4–7]. Previous studies suggested that epigenetic changes, such as microRNAs (miRNAs), histone modifications and DNA methylation, are involved in cancer cell EMT progression [8,9]. MiRNAs are a kind of short non-coding RNA (ncRNA) that degrade mRNAs and suppress protein expression [10]. In non-small cell lung cancer, the ectopic expression of miR-138 inhibits the EMT progression and cancer cell invasion [11]. Sun *et al*. reported that miR-138 modulates metastatic potential in bladder cancer cells by targeting ZEB2 [12].

The article "Long non-coding RNA LINC00152 promotes gallbladder cancer metastasis and epithelial–mesenchymal transition by regulating HIF-1α via miR-138" was retracted in 2023. Reasons: manipulated images; duplicated images; unreliable data; unreliable results or conclusions.

Long non-coding RNAs (lncRNAs) represent a class of ncRNAs longer than 200 nucleotides that lack protein-coding potential [13]. The regulatory function of lncRNAs is very extensive, including chromatin modulation, gene transcription, post-transcriptional modulation, protein function or localization and intercellular signalling [14,15]. LINC00152, a 828 bp lncRNA that maps to chromosome 2p11.2, was initially detected as differentially hypomethylated during hepatocarcinogenesis [16]. Zhao *et al.* reported that LINC00152 is involved in the EMT progression and promotes metastasis in gastric cancer [17]. Our previous studies found that the lncRNAs H19 and MINCR contribute to cell invasion and metastasis via regulating EMT in GBC [4,7]. In this study, we demonstrate that LINC00152 functions as a competing endogenous RNA (ceRNA) for miR-138. The sponging of miR-138 by LINC00152 overexpression has oncogenic effects as miR-138 is no longer able to suppress the downstream target hypoxia inducible factor-1α (HIF-1α) that is involved in GBC metastasis.

## 2. Material and methods

### 2.1. Patients and samples

Thirty-five GBC tissue samples and neighbouring non-cancerous gallbladder tissue samples were obtained from patients who had undergone surgery from April 2009 to February 2012 in Xinhua Hospital (Shanghai, China). Each sample was snap-frozen in liquid nitrogen and stored at −80°C prior to RNA isolation. Each sample was reviewed by two pathologists. None of the patients recruited to this study had received any pre-operative treatments. GBC patients were staged according to the tumour node metastasis staging system (the 7th edition) of the American Joint Committee on Cancer (AJCC). Complete clinicopathological follow-up data of the GBC patients were available.

### 2.2. Cell culture

The immortalized human non-tumorigenic biliary epithelial cell line (H69) and GBC cell lines (GBC-SD, NOZ) were used in this study. GBC-SD and H69 were purchased from the cell bank of the Chinese Academy of Science (Shanghai, China). NOZ was purchased from the Health Science Research Resources Bank (Osaka, Japan). GBC-SD was cultured in DMEM high-glucose medium (Gibco, USA), NOZ was cultured in Williams's Medium E (Genom, China) supplemented with 10% fetal bovine serum (Gibco, USA) at 37°C in a humidified incubator with the presence of 5% CO_2_. Hypoxia (1% O_2_, 5% CO_2_ and 94% N_2_) treatments were carried out in a Forma 0125/1029 Anaerobic Chamber (Thermo Scientific, USA).

The article "Long non-coding RNA LINC00152 promotes gallbladder cancer metastasis and epithelial–mesenchymal transition by regulating HIF-1α via miR-138" was retracted in 2023. Reasons: manipulated images; duplicated images; unreliable data; unreliable results or conclusions.

### 2.3. Total RNA extraction, reverse transcription and qPCR

Total RNA was extracted from GBC tissue samples and cell lines using TRIzol (TaKaRa, China) according to the manufacturer's protocol. For mRNA and lncRNA analyses, the reverse transcription and qPCR reactions were performed as previously described [18]. ACTIN was used as an internal control. For miRNA analyses, RNA was reversed transcribed into cDNAs using the microRNA First Strand cDNA Synthesis kit (Sangon Biotech, China). The cDNA template was amplified by real-time RT-PCR using the microRNAs Quantitation PCR kit (Sangon Biotech, China). Expression of miRNA was normalized with respect to small nuclear RNA U6. The real-time PCRs were performed in triplicate. The relative mRNA expression change was calculated by using 2^−△△Ct^ method. The PCR primers used were as follows: 5′-AAAGACCTGTACGCCAACAC-3′ (forward) and 5′-GTCATACTCCTGCTTGCTGAT-3′ (reverse) for ACTIN, 5′-TGGGAATGGAGGGAAATAAA-3′ (forward) and 5′-CCAGGAACTGTGCTGTGAAG-3′ (reverse) for LINC00152, and 5′-TGCAACATGGAAGGTATTGC-3′ (forward) and 5′-TTCACAAATCAGCACCAAGC-3′ (reverse) for HIF-1α.

### 2.4. RNAi and transfection

Two LINC00152-siRNAs, two HIF-1α-siRNAs and their negative control (NC) siRNAs, plasmids pPG-miR-eGFP-Blasticidin with hsa-miR-138 mimics (pPG-miR-138) or hsa-miR-138 inhibitor (pPG-anti-miR-138) or their NC (pPG-miR-NC), were purchased from GenePharma, China. The sequences of siRNAs are listed as follows: 5′-GGAAUGCAGCUGAAAGAUUTT-3′ (sense) and 5′-AAUCUUUCAGCUGCAUUCCTT-3′ (antisense) for si-LINC00152–1, 5′-GGUGGUCUGCCUGUGAUAUTT-3′ (sense) and 5′-AUAUCACAGGCAGACCACCTT-3′ (antisense) for si-LINC00152-2, 5′-AGAACCCAUUUUCUACUCAGTT-3′ (sense) and 5′-CUGAGUAGAAAAUGGGUUCUTT-3′ (antisense) for si-HIF-1α-1, 5′-GACACAGCCUGGAUAUGAATT-3′ (sense) and 5′-UUCAUAUCCAGGCUGUGUCTT-3′ (antisense) for si-HIF-1α-2, and 5′-UUCUCCGAACGUGUCACGUTT-3′ (sense) and 5′-ACGUGACACGUUCGGAGAATT-3′ (antisense) for NC siRNA. The pcDNA3.1-LINC00152 and the empty vector were purchased from Sangon Biotech, China. Cells were cultured on six-well plates to confluency and transfected with siRNAs or plasmids using Lipofectamine 2000 (Invitrogen, USA) according to the manufacturer's protocol. After 48 h, cells were harvested for the subsequent experiments.

The article "Long non-coding RNA LINC00152 promotes gallbladder cancer metastasis and epithelial–mesenchymal transition by regulating HIF-1α via miR-138" was retracted in 2023. Reasons: manipulated images; duplicated images; unreliable data; unreliable results or conclusions.

### 2.5. Wound healing assay

About 1 × 10^6^ cells were seeded into six-well plates and incubated at 37°C until cells reached a confluence of at least 90%. Wounds were created by scratching cell monolayers with a 200 µl plastic pipette tip and then incubated in fresh medium containing 1% fetal calf serum for 24 h. Photographs were taken to estimate the mean number of migrating cells per field.

### 2.6. Transwell invasion assay

Cell invasion assays were performed using 24-well transwell plates (Corning, USA) pre-coated with Matrigel (BD, USA). About 2 × 10^5^ cells were seeded in the upper chamber with serum free medium in triplicate. Medium containing 10% fetal bovine serum (300 µl) was added to the lower chamber as chemo-attractant. After incubation for 24 h, the cells above the Matrigel layer were removed by cotton swab, and the cells below the membrane were fixed by methanol, stained with 0.1% crystal violet for 10 min, and counted from five randomly chosen fields for each well.

### 2.7. Dual-luciferase reporter assay

NOZ Cells were co-transfected with 150 ng of empty pmiR-GLO-NC, pmiR-GLO-LINC00152-wt or pmiR-GLO-LINC00152-mut, pmiR-GLO-HIF-1α-wt or pmiR-GLO-HIF-1α-mut (Sangon Biotech, China), and 2 ng of internal control pRL-TK (Promega, USA). pPG-miR-138 or pPG-miR-NC were also co-transfected into NOZ cells. HIF-1α siRNA or its control (si-NC) was co-transfected with Slug promoter construct pGL3-Slug or its control pGL3-control (Sangon Biotech, China) and internal control pRL-TK into NOZ cells. The luciferase activities were assessed using a dual-luciferase reporter assay kit (Promega, USA) according to the manufacturer's protocol. The relative luciferase activity was normalized to Renilla luciferase activity.

### 2.8. RNA-binding protein immunoprecipitation assay

RNA immunoprecipitation (RIP) assays were performed using the EZ-Magna RIP RNA-Binding Protein Immunoprecipitation Kit (Millipore, USA) according to the manufacturer's protocol. NOZ cells were lysed in complete RIP lysis buffer and cleared lysates were then incubated with RIP buffer containing magnetic beads conjugated to human anti-Ago2 antibody (Proteintech, China). The NC was normal mouse IgG (Beyotime, China), and the positive control was SNRNP70 (Millipore, USA). The coprecipitated RNAs were isolated by TRIzol reagent (TaKaRa, China) and were detected by qPCR.

### 2.9. Biotin-labelled miRNA pull-down assay

NOZ cells were transfected with biotinylated miR-138, biotinylated miR-138-mut and biotinylated NC (GenePharma, China). Cells were collected at 48 h. The cell lysates were incubated with M-280 streptavidin magnetic beads (Invitrogen, USA). To prevent non-specific binding of RNA and protein complexes, the beads were coated with RNase-free bovine serum albumin and yeast tRNA (both from Sigma-Aldrich). The beads were incubated at 4°C for 3 h, and washed three times with ice-cold lysis buffer and once with high salt buffer (0.1% SDS, 1% Triton X-100, 2 mM EDTA, 20 mM Tris–HCl, pH 8.0 and 500 mM NaCl). The bound RNAs were purified using TRIzol for the analysis.

The article "Long non-coding RNA LINC00152 promotes gallbladder cancer metastasis and epithelial–mesenchymal transition by regulating HIF-1α via miR-138" was retracted in 2023. Reasons: manipulated images; duplicated images; unreliable data; unreliable results or conclusions.

### 2.10. Lentiviral transfection for stable LINC00152 expression

LV3-pGLV-H1-GFP + Puro plasmids with pcDNA-LINC00152 or control oligonucleotides, namely LV-LINC00152 and LV-NC, were purchased from GenePharma, China. Lentivirus transfections were performed according to the manufacturer's protocol to establish the stable LINC00152-expressing GBC-SD cells (GBC-SD/LV-LINC00152). The control clones (GBC-SD/LV-NC) were constructed similarly. The expression level of LINC00152 was assessed by qPCR.

### 2.11. Immunofluorescence analysis

Cells were grown on glass coverslips in a six-well plate and then fixed in a solution of 4% paraformaldehyde in PBS for 30 min. The cells were permeabilized with 0.1% Triton X-100 in PBS for 15 min, and blocked in 5% goat serum in PBS for 1 h. Coverslips were then incubated in primary antibodies overnight at 4°C with the following dilutions: E-cadherin and Vimentin (1 : 50, Santa Cruz, USA), Slug (1 : 400, Cell Signaling Technology, USA). Cells were washed and incubated in secondary antibody (Abcam, USA) for 1.5 h at 37°C. Immunofluorescence was analysed using fluorescence microscopy (Olympus BX51).

### 2.12. Western blot

Western blot assay was carried out as previously described [18]. Total protein was extracted with RIPA lysis buffer (Solarbio, China) supplemented with protease inhibitors (Roche Applied Science, Switzerland). The primary antibodies used were anti-E-cadherin (1 : 500, Santa Cruz, USA), anti-Vimentin (1 : 500, Santa Cruz, USA), anti-Twist (1 : 500, Santa Cruz, USA), anti-HIF-1α (1 : 500, Proteintech, China), anti-Slug (1 : 1000, Cell Signaling Technology, USA), anti-Snail (1 : 1000, Cell Signaling Technology, USA), anti-MMP2 (1 : 1000, Cell Signaling Technology, USA), anti-MMP9 (1 : 1000, Cell Signaling Technology, USA) and anti-GAPDH (1 : 5000, Proteintech, China). Horseradish peroxidase-conjugated goat anti-mouse or goat anti-rabbit IgG antibody (1 : 1000, Beyotime, China) was used as secondary antibodies. All experiments were performed in triplicate.

### 2.13. Tumour peritoneal metastasis

All animal experiments were performed in the animal laboratory centre of Ruijin Hospital of Shanghai JiaoTong University School of Medicine (Shanghai, China). The study protocol was approved by the Animal Care and Use committee of Ruijin Hospital. GBC-SD cells transfected with LV-LINC00152 or LV-NC were intraperitoneally injected into each four-week-old male nude mouse (three mice for each group). After 35 days, mice were sacrificed and peritoneal metastatic nodules were calculated.

The article "Long non-coding RNA LINC00152 promotes gallbladder cancer metastasis and epithelial–mesenchymal transition by regulating HIF-1α via miR-138" was retracted in 2023. Reasons: manipulated images; duplicated images; unreliable data; unreliable results or conclusions.

### 2.14. Statistical analysis

All statistical analyses were performed using SPSS 20.0 (SPSS, USA). The expression level of LINC00152 in tumour tissue samples was compared with adjacent non-tumour tissue samples using paired-samples *t*-test. The differences between groups were analysed using independent-samples *t*-test. All data are presented as mean ± s.d. All the *p*-values were two-sided and *p* < 0.05 was deemed statistically significant.

## 3. Results

### 3.1. LINC00152 is significantly upregulated in gallbladder cancer and associated with clinicopathologic characteristics

First, we performed qPCR to assess the expression levels of LINC00152 in 35 pairs of GBC tissue samples and paired adjacent normal tissue samples. As shown in figure 1*a*, LINC00152 levels in GBC tissue samples were significantly higher than those in paired adjacent normal tissue samples. Similarly, LINC00152 levels were upregulated in two GBC cell lines (GBC-SD and NOZ) compared with human normal biliary epithelial H69 cells (figure 1*b*). Furthermore, we found that high LINC00152 expression group (*n* = 18, LINC00152 expression ratio ≥ median ratio) has shorter overall survival time than low LINC00152 expression group (*n* = 17, LINC00152 expression ratio < median ratio) (figure 1*c*). As indicated in table 1, the expression level of LINC00152 was correlated positively with tumour status progression (*p* = 0.027) and lymph node invasion (*p* = 0.028). Nonetheless, there was no significant association between the LINC00152 expression and gender, age, histological grade and clinical stage. Together, these data indicate that increased LINC00152 expression might be related to GBC progression.

**Figure 1.** LINC00152 is overexpressed in GBC tissue samples. (*a*) LINC00152 expression levels in GBC and adjacent normal tissue samples were detected by qPCR (*n* = 35). The relative expression fold change of mRNAs was calculated by the 2^−△△Ct^ method. The expression of LINC00152 was normalized to ACTIN. The statistical differences between samples were analysed with paired-samples *t*-test. (*b*) LINC00152 expression levels in GBC cell lines NOZ and GBC-SD were detected by qPCR and compared with those in the human gallbladder epithelium cell line H69. The expression of LINC00152 was normalized to that in H69. (*c*) LINC00152 correlates negatively with overall survival time (log-rank = 4.331, *p* < 0.05). The mean ± s.d. of triplicate experiments were plotted, ***p < 0.001.

The article "Long non-coding RNA LINC00152 promotes gallbladder cancer metastasis and epithelial–mesenchymal transition by regulating HIF-1α via miR-138" was retracted in 2023. Reasons: manipulated images; duplicated images; unreliable data; unreliable results or conclusions.

**Table 1.** The association of LINC00152 expression in 35 GBC patients with clinicopathologic characteristics.

characteristics	case number	LINC00152 expression		*p*-value
		low (*n* = 17)	high (*n* = 18)	
gender				0.208
male	9	6	3	
female	26	11	15	
age				0.404
≤60	16	9	7	
>60	19	8	11	
histological grade				0.227
well and moderately	11	7	4	
poorly and others	24	10	14	
T status				0.027*
T1–2	14	10	4	
T3–4	21	7	14	
N status				0.028*
N0	18	12	6	
N1/2	17	5	12	
clinical stage				0.105
I–II	13	4	9	
III–IV	22	13	9	

*p < 0.05.

### 3.2. Reciprocal repression of LINC00152 and miR-138 in gallbladder cancer cell

To further explore the function of LINC00152 in GBC, we transfected GBC-SD cells with plasmids containing pcDNA-LINC00152 or pcDNA-NC and NOZ cells with LINC00152-siRNAs or NC. The overexpressing and interfering efficiency were confirmed by qPCR (figure 2*a,b*). We selected si-LINC00152-1 in the subsequent assays for its more effective inhibition.

**Figure 2.** Identification of miR-138 as a target of LINC00152. (*a*) The expressions of LINC00152 in cell line GBC-SD transfected with pcDNA-LINC00152 or pcDNA-NC were quantified by qPCR. (*b*) The expressions of LINC00152 in cell line NOZ transfected with two different siRNAs against LINC00152 or si-NC were quantified by qPCR. (*c*) Alignment of miR-138 sequence with LINC00152 and with LINC00152 mutated at the putative binding site. (*d,e*) The expression of miR-138 was upregulated after silencing LINC00152 in NOZ cells and downregulated after overexpressing LINC00152 in GBC-SD cells. (*f*) miR-138 is downregulated in GBC tissue samples compared with levels in adjacent normal tissue samples as determined by qPCR. The expression of miR-138 was normalized to U6. (*g*) The correlation between LINC00152 expression level and miR-138 level was measured in 35 GBC tissue samples (*r* = −0.407, *p* < 0.05). The △Ct values were subjected to Pearson's correlation analysis. (*h*,*i*) The expressions of miR-138 in NOZ and GBC-SD cells transfected with pPG-miR-138, pPG-anti-miR-138 or pPG-miR-NC were quantified by qPCR. (*j,k*) The expressions of LINC00152 in NOZ and GBC-SD cells transfected with pPG-miR-138, pPG-anti-miR-138 or pPG-miR-NC were quantified by qPCR. The mean ± s.d. of triplicate experiments were plotted. **p < 0.01, ***p < 0.001.

Through being like a molecular sponge or ceRNA, lncRNAs could competitively interact with their same miRNA responsive elements and then regulate the protein expression [19]. Chen *et al*. [20] demonstrated that LINC00152 is present in both nucleus and cytoplasm. We hypothesized that LINC00152 could function as a molecular sponge and modulate miRNAs in cytoplasm. Through prediction in online databases (miRcode, http://www.mircode.org/index.php), we found that there are putative complementary sequences between LINC00152 and miR-138. The putative binding site is presented in figure 2*c*. Interestingly, our previous study demonstrated that miR-138 is significantly downregulated and suppresses cell proliferation in GBC [21]. Then we performed qPCR to detect the expression levels of miR-138 in si-LINC00152 transfected NOZ cells and pcDNA-LINC00152 transfected GBC-SD cells. As we expected, the expression of miR-138 showed a significant increase in NOZ/si-LINC00152 and decrease in GBC-SD/pcDNA-LINC00152 compared with their NC groups (figure 2*d,e*).

The article "Long non-coding RNA LINC00152 promotes gallbladder cancer metastasis and epithelial–mesenchymal transition by regulating HIF-1α via miR-138" was retracted in 2023. Reasons: manipulated images; duplicated images; unreliable data; unreliable results or conclusions.

In addition, we performed qPCR to assess the expression levels of miR-138 in the 35 GBC patients and confirmed its downregulation in GBC tissue samples, while its levels correlated negatively with LINC00152 levels (*r* = −0.407, *p* < 0.05, figure 2*f,g*). To further determine that whether miR-138 is capable of negatively regulating LINC00152, we transfected GBC cells with pPG-miR-138, pPG-anti-miR-138 or pPG-miR-NC. The qPCR results showed that pPG-anti-miR-138 significantly reduced the endogenous miR-138 and increased LINC00152 expression, while pPG-miR-138 dramatically increased the miR-138 level and suppressed LINC00152 expression in NOZ and GBC-SD cells (figure 2*h–k*).

### 3.3. LINC00152 directly binds to miR-138

MiRNAs exert their miRNA-mediated gene silencing function by binding to Ago2, a core component of the RNA-induced silencing complex (RISC) [22]. We performed RIP assays with Ago2 antibody to isolate the RNA from RISC. The result indicated that LINC00152 was preferentially enriched in Ago2-containing beads in NOZ cells (figure 3*a*). Moreover, we performed miRNA pull-down assays by transfecting biotinylated miR-138, biotinylated miR-138-mut or biotinylated NC into NOZ cells. We observed that LINC00152 could be pulled down by miR-138 (figure 3*b*). And we demonstrated that LINC00152 could directly bind to miR-138.

**Figure 3.** The underlying mechanism of the regulation of miR-138 and LINC00152. (*a*) Amount of LINC00152 bound to SNRNP70 (a positive control), Ago2 or IgG (a negative control) was measured by qPCR after RIP in NOZ cells. (*b*) NOZ cells were transfected with biotinylated NC (Bio-NC), biotinylated wild-type miR-138 (Bio-miR-138) or biotinylated mutant miR-138 (Bio-miR-138-mut), and biotin-based miRNA pull-down assays were conducted after 48 h of transfection. LINC00152 levels were analysed by qPCR. (*c*) Luciferase reporter activity in NOZ cells was detected after co-transfection with pPG-miR-138 (or the empty vector as a control) and the luciferase empty vector (pmiR-GLo), or the vector containing the wild-type LINC00152 (pmiR-GLo-LINC00152-wt) or mutant transcripts (pmiR-GLo-LINC00152-mut). Data are presented as the relative ratio of firefly luciferase activity to Renilla luciferase activity. (*d*) Luciferase reporter activity in NOZ cells was detected after co-transfection with pPG-miR-138 (or the empty vector as a control) and the luciferase empty vector (pmiR-GLo), or the vector containing the wild-type HIF-1α (pmiR-GLo-HIF-1α-wt) or mutant transcripts (pmiR-GLo-HIF-1α-mut). Data are presented as the relative ratio of firefly luciferase activity to Renilla luciferase activity. The mean ± s.d. of triplicate experiments were plotted. **p < 0.01, ***p < 0.001; n.s., not statistically significant.

The article "Long non-coding RNA LINC00152 promotes gallbladder cancer metastasis and epithelial–mesenchymal transition by regulating HIF-1α via miR-138" was retracted in 2023. Reasons: manipulated images; duplicated images; unreliable data; unreliable results or conclusions.

To further explore whether the binding site is functional, a dual-luciferase reporter assay in NOZ cells was carried out. The luciferase activity was reduced in cells co-transfected with pPG-miR-138 + pmiR-Glo-LINC00152-wt but not in cells co-transfected with pPG-miR-138 + pmiR-Glo or pPG-miR-138 + pmiR-Glo-LINC00152-mut (figure 3*c*). These data suggest that the binding site is essential for the reciprocal repression of LINC00152 and miR-138.

### 3.4. LINC00152 positively regulates HIF-1α, a target of miR-138

Yeh *et al*. [23] and Song *et al*. [24] reported that HIF-1α is a target of miR-138. Here we observed the similar phenomenon of mRNA and protein level changes in GBC cells (figure 4*a,b*). Furthermore, we constructed wild-type and mutated luciferase reporters of HIF-1α. And the results of luciferase reporter assays confirmed that there is a direct interaction between miR-138 and the 3′UTR of HIF-1α in NOZ cells (figure 3*d*). Then we explored whether LINC00152 could regulate HIF-1α by competing with miR-138 in GBC cell lines. Knockdown of LINC00152 in NOZ cells dramatically inhibited HIF-1α mRNA and protein expression levels while pPG-anti-miR-138 reversed these effects (figure 4*c,d*). Conversely, when we amplified LINC00152 expression in GBC-SD cells, the HIF-1α mRNA and protein expression levels was significantly upregulated, and pPG-miR-138 reversed these effects (figure 4*e,f*). These data indicate that LINC00152 positively regulates HIF-1α, at least in part, through binding miR-138.

**Figure 4.** HIF-1α is regulated by miR-138 and LINC00152. (*a,b*) The mRNA and protein levels of HIF-1α in NOZ cells transfected with pPG-miR-138, pPG-anti-miR-138 or pPG-miR-NC were measured by qPCR and western blot assays. (*c,d*) The mRNA and protein levels of HIF-1α in NOZ cells transfected with si-NC, si-LINC00152 or si-LINC00152 + pPG-anti-miR-138 were measured by qPCR and western blot assays. (*e,f*) The mRNA and protein levels of HIF-1α in GBC-SD cells transfected with pcDNA-NC, pcDNA-LINC00152 or pcDNA-LINC00152 + pPG-miR-138 were measured by qPCR and western blot assays. The mean ± s.d. of triplicate experiments were plotted. **p < 0.01; n.s., not statistically significant.

The article "Long non-coding RNA LINC00152 promotes gallbladder cancer metastasis and epithelial–mesenchymal transition by regulating HIF-1α via miR-138" was retracted in 2023. Reasons: manipulated images; duplicated images; unreliable data; unreliable results or conclusions.

### 3.5. LINC00152 promotes gallbladder cancer cell metastasis and epithelial–mesenchymal transition progression

To explore the role of LINC00152 in GBC cell metastasis, we performed the wound healing and transwell invasion assays to assess the effect of LINC00152 knockdown/overexpression on cell migration and invasion ability. Compared with control cells, LINC00152 knockdown in NOZ cells significantly decreased cell migration and invasion, while LINC00152 overexpression in GBC-SD cells significantly promoted cell migration and invasion (figures 5*d–g* and 6). Therefore, the role of LINC00152 in promoting GBC cell metastasis is functional. It is well known that extracellular matrix degradation by matrix metalloproteinases (MMPs) such as MMP2 and MMP9 plays an important role in GBC migration and invasion [25–27]. Also, we found that the expression of MMP9 was decreased in si-LINC00152 NOZ cells, but not MMP2 (figure 5*c*).

**Figure 5.** Knockdown of LINC00152 or HIF-1α inhibits GBC cell migration and invasion. (*a,b*) The mRNA and protein levels of HIF-1α in NOZ cells transfected with two different siRNAs against HIF-1α or si-NC were quantified by qRT-PCR and western blot assays. (*c*) The protein levels of MMP2 and MMP9 in NOZ cells transfected with si-LINC00152 or si-NC were measured by western blot assay. (*d,f*) Wound healing assays in NOZ cells transfected with si-NC, si-HIF-1α, si-LINC00152 or si-LINC00152 + pPG-anti-miR-138 are shown. (*e,g*) Transwell invasion assays in NOZ cells transfected with si-NC, si-HIF-1α, si-LINC00152 or si-LINC00152 + pPG-anti-miR-138 are shown. The mean ± s.d. of triplicate experiments were plotted. **p < 0.01, ***p < 0.001; n.s., not statistically significant.

**Figure 6.** Ectopic expression of LINC00152 promotes GBC cell migration and invasion. (*a,c*) Wound healing assays in GBC-SD cells transfected with pcDNA-NC, pcDNA-LINC00152 or pcDNA-LINC00152 + pPG-miR-138 are shown. (*b,d*) Transwell invasion assays in NOZ cells transfected with pcDNA-NC, pcDNA-LINC00152 or pcDNA-LINC00152 + pPG-miR-138 are shown. The mean ± s.d. of triplicate experiments were plotted. **p < 0.01, ***p < 0.001; n.s., not statistically significant.

The article "Long non-coding RNA LINC00152 promotes gallbladder cancer metastasis and epithelial–mesenchymal transition by regulating HIF-1α via miR-138" was retracted in 2023. Reasons: manipulated images; duplicated images; unreliable data; unreliable results or conclusions.

To explore whether LINC00152 regulates GBC cell metastasis through inducing EMT, we next performed immunofluorescence and western blot assays to assess the expression levels of an epithelial marker, E-cadherin, and of a mesenchymal marker, Vimentin, in LINC00152 knockdown/overexpression GBC cell. As shown in figure 7, LINC00152 knockdown could increase E-cadherin expression and decrease Vimentin expression in NOZ cells, while the opposite results were obtained after LINC00152 was overexpressed in GBC-SD cells. These results suggested that LINC00152 is capable of potentiating the epithelial cells to transdifferentiate into mesenchymal cells.

**Figure 7.** LINC00152 promotes GBC cell EMT progression. (*a,b*) The protein levels of Vimentin and E-cadherin in NOZ cells transfected with si-NC, si-LINC00152 or si-HIF-1α were measured by immunofluorescence and western blot assays. (*c,d*) The protein levels of Vimentin and E-cadherin in GBC-SD cells transfected with pcDNA-NC or pcDNA-LINC00152 were measured by immunofluorescence and western blot assays.

### 3.6. MiR-138 inhibits gallbladder cancer cell metastasis and epithelial–mesenchymal transition progression

Previous studies reported that miR-138 suppresses cell metastasis and EMT progression in various types of cancer [11,28,29]. However, its role in GBC had not been elucidated. In this part, we demonstrated that the effect of miR-138 on GBC cell migration, invasion and EMT was opposite to that of LINC00152 (figures 8 and 9). In addition, we also co-transfected LINC00152 knockdown NOZ cells with pPG-anti-miR-138 and LINC00152 overexpressing GBC-SD cells with pPG-miR-138, and the number of migrating and invading cells was significantly reversed for both (figures 5*d–g* and 6).

**Figure 8.** miR-138 inhibits GBC cell migration and invasion. (*a,c*) Wound healing assays in NOZ cells transfected with pPG-miR-138, pPG-anti-miR-138 or pPG-miR-NC are shown. (*b,d*) Transwell invasion assays in NOZ cells transfected with pPG-miR-138, pPG-anti-miR-138 or pPG-miR-NC are shown. The mean ± s.d. of triplicate experiments were plotted. **p < 0.01; n.s., not statistically significant.

**Figure 9.** miR-138 promotes GBC cell EMT progression. (*a,b*) The protein levels of Vimentin and E-cadherin in NOZ cells transfected with pPG-miR-138, pPG-anti-miR-138 or pPG-miR-NC were measured by immunofluorescence and western blot assays.

### 3.7. Knockdown of HIF-1α inhibits gallbladder cancer cell metastasis and epithelial–mesenchymal transition progression

Many studies on human malignant neoplasms have reported that HIF-1α induces cell metastasis and EMT progression in cancer cells [30–35]. However, the role of HIF-1α in GBC cell metastasis and EMT progression had never been elucidated before. To stop HIF-1α expression in GBC cells, we transfected two HIF-1α-specific siRNAs into NOZ cells. As shown in figure 5*a,b*, interference of HIF-1α mRNA and protein levels was observed in si-HIF-1α-2 cells, and we chose this siRNA for HIF-1α knockdown.

The article "Long non-coding RNA LINC00152 promotes gallbladder cancer metastasis and epithelial–mesenchymal transition by regulating HIF-1α via miR-138" was retracted in 2023. Reasons: manipulated images; duplicated images; unreliable data; unreliable results or conclusions.

As wound healing and transwell invasion assays indicated, HIF-1α knockdown dramatically inhibited cell migration and invasion in NOZ cells (figure 5*d–g*). Additionally, the immunofluorescence and western blot analyses showed that the expression of Vimentin was related to HIF-1α expression, but opposite to E-cadherin, which suggested that HIF-1α might be involved in regulating EMT progression of GBC cell (figure 7*a,b*).

Some previous studies reported that HIF-1α is capable of promoting EMT progression by activating some direct EMT regulators such as Slug, Snail and Twist [36–38]. To further explore the mechanism of HIF-1α on the regulation of EMT progression in GBC, we transfected NOZ cells with si-LINC00152 or si-HIF-1α and assessed the expression levels of HIF-1α, Slug, Snail and Twist under hypoxia conditions. As shown in figure 10*a*, we confirmed that LINC00152 knockdown could significantly decrease the expression of HIF-1α under hypoxia conditions. As to the three EMT regulators, either knockdown of LINC00152 or HIF-1α decreased the expression of Slug in NOZ cells under hypoxia conditions, but not Snail and Twist (figure 10*a,b*). We considered that Slug may be a downstream mediator of LINC00152/miR-138/HIF-1α pathway in GBC cell EMT progression. Next, we cloned Slug promoter (−2000 to 0 bp) into the pGL3 basic luciferase reporter, and co-transfected it with si-HIF-1α into NOZ cells under hypoxia conditions. Consistent with the western blot results above, figure 10*c,d* indicate the luciferase activity of Slug promoter was significantly decreased in HIF-1α knockdown NOZ cells.

**Figure 10.** Slug is a direct target of HIF-1α in GBC. (*a*) The protein levels of HIF-1α, Slug, Snail and Twist in NOZ cells transfected with si-LINC00152, si-HIF-1α or si-NC under hypoxia conditions were measured by western blot assay. (*b*) The protein levels of Slug in NOZ cells transfected with si-HIF-1α, si-LINC00152 or si-NC under hypoxia conditions were measured by immunofluorescence assay. (*c*) Luciferase reporter assay in NOZ cells was detected after transfection with firefly luciferase constructs containing the Slug promoter (−2000 to 0 bp) or the luciferase empty vector under hypoxia or normoxia conditions. Data are presented as the relative ratio of firefly luciferase activity to Renilla luciferase activity. (*d*) Luciferase reporter assay in NOZ cells was detected after co-transfection with firefly luciferase constructs containing the Slug promoter (−2000 to 0 bp) or the luciferase empty vector and si-HIF-1α or si-NC under normoxia conditions. Data are presented as the relative ratio of firefly luciferase activity to Renilla luciferase activity. The mean ± s.d. of triplicate experiments were plotted. **p < 0.01, ***p < 0.001; n.s., not statistically significant.

The article "Long non-coding RNA LINC00152 promotes gallbladder cancer metastasis and epithelial–mesenchymal transition by regulating HIF-1α via miR-138" was retracted in 2023. Reasons: manipulated images; duplicated images; unreliable data; unreliable results or conclusions.

### 3.8. LINC00152 promotes gallbladder cancer cell peritoneal spreading and metastasis *in vivo*

Finally, to investigate the effect of LINC00152 on tumour metastasis *in vivo*, we injected GBC-SD cells with LV-LINC00152 or LV-NC into nude mice intraperitoneally. A nearly 300-fold LINC00152 increase was observed in GBC-SD/LV-LINC00152 cells (figure 11*a*). Five weeks after injection, the number of intraperitoneal metastatic nodules derived from the GBC-SD/LV-LINC00152 group was significantly more than that derived from the control group (7.33 ± 1.52 versus 16.33 ± 3.06, *p* < 0.05; figure 11*b,c*). Thus, LINC00152 has the capability to promote tumour GBC cell peritoneal spreading and metastasis *in vivo*.

**Figure 11.** Effect of LINC00152 on peritoneal spreading and metastasis *in vivo*. (*a*) The expression of LINC00152 in GBC-SD cells transfected with LV-LINC00152 and LV-NC were quantified by qPCR. (*b,c*) The number of the peritoneal spreading and metastasis nodules derived from GBC-SD/LV-LINC00152 and GBC-SD/LV-NC in nude mice was evaluated. The mean ± s.d. of triplicate experiments were plotted. *p < 0.05, ***p < 0.001.

## 4. Discussion

Some recent studies had shown that LINC00152 is overexpressed in multiple tumour types and the upregulation is able to enhance tumour metastasis [17,20]. In this study, we collected a considerable number of GBC patients, and found that LINC00152 is also aberrantly upregulated in GBC and the high LINC00152 level is negatively correlated with the overall survival time. By manipulating LINC00152 expression, we observed its positive effects on GBC cell migration, invasion and EMT *in vitro*, while the peritoneal spreading and metastasis assay confirmed these effects *in vivo*. Thus, we believe that LINC00152 potentiates the aggression and metastasis of GBC by acting as an inducer of EMT. Next, we tried to elucidate the mechanism by which LINC00152 overexpression promotes tumour metastasis and EMT progression.

Five years ago, Salmena *et al*. [19] first proposed a hypothesis that ceRNA activity may play vital roles in human cancers by forming an extensive regulatory network across the transcriptome, thereby extremely expanding the functional genetic information. The ceRNA network often presents a reciprocal repression between lncRNAs and miRNAs. Accumulating evidence suggested that lncRNAs might compete for endogenous miRNAs by the binding of their same response elements and affect the target genes of miRNAs. It has been shown that ZFAS1 promotes hepatocellular carcinoma metastasis by modulating ZEB1, MMP14 and MMP16, and sponging miR-150 [39]. Moreover, the lncRNA APF was also shown to regulate autophagic cell death and myocardial infarction by regulating ATG7 as a ceRNA for miR-188-3p in cardiovascular diseases [40]. LINC00152 is a relatively new lncRNA, and little is known about its ‘sponge’ role for miRNAs. Chen *et al*. [20] demonstrated that LINC00152 was present in both cytoplasm and nucleus of gastric cancer cells, and it could bind to enhancer of zeste homologue 2 in nucleus. Therefore, we asked whether LINC00152 targets miRNAs in cytoplasm of GBC cell. We observed that LINC00152 knockdown upregulated miR-138 and LINC00152 overexpression suppressed miR-138, which could repress cell migration, invasion and EMT progression in GBC. Our previous study has shown that miR-138 is downregulated in GBC [21], and our present study confirmed that its expression is downregulated and correlates negatively with LINC00152 expression in the 35 GBC patients. The reciprocal repression between lncRNAs and miRNAs has often been observed. Through a two-step processing, mature miRNAs are produced by Drosha and Dicer [41]. The initial process occurs in the nucleus when pri-miRNA is cleaved into pre-miRNA by Drosha-DGCR8 complex. The second processing step occurs in the cytoplasm such that Dicer complex cleaves pre-miRNA into a mature miRNA duplex [42]. We supposed that the effect of LINC00152 on miR-138 was through the interaction with Drosha or Dicer. Conversely, our study also demonstrated that LINC00152 could be negatively regulated by miR-138. As miRNAs are known to post-transcriptionally suppress gene expression by interacting with the 3′-untranslated regions of target genes, we supposed that miR-138 promoting the downregulation of LINC00152 was somewhat similar to the miRNA-mediated silencing of protein-coding genes.

The article "Long non-coding RNA LINC00152 promotes gallbladder cancer metastasis and epithelial–mesenchymal transition by regulating HIF-1α via miR-138" was retracted in 2023. Reasons: manipulated images; duplicated images; unreliable data; unreliable results or conclusions.

Ago2, a core component of RISC, binds to miRNAs, thereby modulating the expression of target genes [43]. To test whether LINC00152 and miR-138 bind in the same RISC that plays a vital role in RNA silencing, we carried out the RIP assay and found that LINC00152 was enriched in Ago2-containing beads. Additionally, we carried out the miRNA pull-down assay and found that LINC00152 could be pulled down by biotin-labelled miR-138 in NOZ cells. The dual-luciferase reporter assay also confirmed that the binding between LINC00152 and miR-138 is functional. Based on the results above, we put forward for the first time that LINC00152 could act as a ceRNA for miR-138 in GBC.

HIF-1α, a hypoxia-responsive protein, is often overexpressed in human cancers because of the intratumoural hypoxia condition or genetic alterations. Krishnamachary *et al*. reported that HIF-1α regulates a variety of genes involved in the colorectal cancer cell EMT progression, such as MMP2, fibronectin 1, vimentin and transforming growth factor α [44]. Similarly, Yeh *et al*. [23] reported that Slug is the downstream molecule of HIF-1α in human ovarian cancer. Our present study demonstrated that Slug, but not Snail or Twist, is the direct target gene of HIF-1α under hypoxia conditions and knockdown of LINC00152 decreased MMP9 expression in GBC. The secretion of MMPs with the capacity of extracellular matrix degradation is a feature of metastatic cancer cells [45]. Slug, a direct inhibitor of E-cadherin, acts as a master regulator of EMT progression [46]. To our knowledge, we are the first to show that HIF-1α enhances GBC cell migration, invasion and EMT progression functionally and mechanically. Also, we observed that LINC00152 correlated positively with the endogenous HIF-1α mRNA and protein expression by acting as a ceRNA for miR-138 in NOZ and GBC-SD cell lines.

In summary, LINC00152 promotes GBC metastasis and EMT progression by functioning as a miRNA sponge to abrogate the endogenous effect of miR-138, which suppresses the expression of HIF-1α. The LINC00152/miR-138/HIF-1α signalling pathway regulatory network may be a novel therapeutic target for GBC. The prognostic value of LINC00152 in GBC should be confirmed in future studies with a large cohort of samples.

## Data accessibility

LINC00152 (*Homo sapiens*) sequences: NCBI Reference Sequence accession NR_024204.1. Mature hsa-miR-138 sequences: miRBase accession MIMAT000430.
